The article "Identification of Key Genes in Nasopharyngeal Carcinoma Based on Bioinformatics Analysis" was retracted in 2023. Reasons: signs of a paper mill; compromised peer review; unreliable results or conclusions.

# Identification of Key Genes in Nasopharyngeal Carcinoma Based on Bioinformatics Analysis

**DOI:** 10.1155/2022/9022700

**Published:** 2022-06-07

**Authors:** Yujie Song, Tao Feng, Wenping Cao, Haiyang Yu, Zeng Zhang

**Affiliations:** Department of Otolaryngology, Zibo Central Hospital, Zibo 255000, Shandong, China

## Abstract

**Objective:**

This study aimed to identify key genes associated with the pathogenesis of nasopharyngeal carcinoma (NPC) by bioinformatics analysis.

**Methods:**

Datasets (GSE13597 and GSE34573) were screened and downloaded from the comprehensive gene expression database (GEO). GEO2R online tool was adopted to analyze microarray data GSE13597 and GSE34573 related to NPC. Volcano plot was generated using Bioconductor in R software. “Pheatmap” was used to draw heatmaps based on the top 10 regulated genes of GSE13597 and GSE34573. GO and KEGG analyses were conducted via online tool DAVID. We uploaded the DEGs of NPC to STRING software and then used Cytoscape software to draw PPI network of DEGs.

**Results:**

216 DEGs were obtained in GSE13597 between patient and control group (111 up-regulated DEGs and 105 down-regulated DEGs). 1101 DEGs were obtained in GSE34573 (470 up-regulated DEGs and 641 down-regulated DEGs). 63 common differential genes were screened named co-DEGs in the two datasets. These DEGs were mainly associated with defense response to bacterium, cell-matrix adhesion, chemokine-mediated signaling pathway, tissue homeostasis, humoral immune response, cilium movement, cilium organization, cilium assembly, and epithelial cilium movement. KEGG pathway enrichment analysis showed that DEGs were mainly involved in viral protein interaction with cytokine and cytokine receptor, salivary secretion, p53 signaling pathway, IL-17 signaling pathway, cell cycle, PI3K-Akt signaling pathway, and ECM-receptor interaction. We identified seven hub genes, including FN1, MMP-10, MUC1, KIF23, CDK1, MUC5B, and MUC5AC.

**Conclusions:**

Seven hub genes, including FN1, MMP-10, MUC1, KIF23, CDK1, MUC5B, and MUC5AC, might be therapeutic potential biomarkers of NPC.

## 1. Introduction

Nasopharyngeal carcinoma (NPC) is a kind of tumor characterized by high malignancy, easy metastasis with high incidence in southern China [1]. Scientists have conducted numerous studies on the pathogenesis, susceptibility, and carcinogenesis of NPC. The occurrence and development of NPC is a process of gradual evolution with the participation of multiple genes, which is related to EBV infection, chemical carcinogens, heredity, and other factors. Because the onset site of NPC is relatively hidden and there is no obvious symptom in the early stage, most patients are difficult to be diagnosed in the early stage. At present, most nasopharyngeal carcinoma is squamous cell carcinoma, and the first choice for the treatment of nasopharyngeal carcinoma is radiotherapy [1–3]. In order to ameliorate life quality of patients, surgery, chemotherapy, and radiotherapy are usually used together. In the past research, the most common research ideas to study differentially expressed genes are molecular targeting and diagnostic markers. For instance, Jiang et al. found that 6-hypermethylated genes were negatively associated with survival in NPC patients [2]. Developments in bioinformatics now provide new methods for the identification of genes associated with cancer development.

The article "Identification of Key Genes in Nasopharyngeal Carcinoma Based on Bioinformatics Analysis" was retracted in 2023. Reasons: signs of a paper mill; compromised peer review; unreliable results or conclusions.

As an efficient and large-scale bioinformation acquisition technology, gene chip can detect and analyze differentially expressed genes (DEGs) between patients and normal humans [4, 5]. The analysis of cancer specific gene expression may provide a new research basis for the occurrence and development of human cancer. In the field of cancer research, microarray can be used to study the heterogeneity of cancer diagnosis and treatment response, so as to find the key genes of cancer in epigenetics, which may become molecular markers of cancer diagnosis and prognosis [6, 7]. The research of gene chip in malignant tumor has attracted a lot of attention in recent ten years. Liu et al. identified the histological specific biomarkers of miRNAs-mRNAs related to NPC based on the comprehensive analysis of miRNAs and mRNAs microarray. The results showed that miR-452-ITGA9 was obviously related to the survival rate of NPC invalids [8].

Present study used bioinformatics analysis to screen the related DEGs from NPC and normal nasopharyngeal tissues. Then, we conducted cluster and functional enrichment analysis of DEGs. The protein-protein interaction (PPI) network was found to further screen the hub genes. Finally, seven hub genes were obtained via intersection of two datasets, which can provide potential biomarkers for NPC for follow-up research.

## 2. Material and Methods

### 2.1. Data Sources

We first entered the keywords “nasopharyngeal carcinoma” and “*Homo sapiens*” in the search box of the geo database website (https://www.ncbi.nlm.nih.gov/geo/) and selected keyword for retrieval. According to the search results, we obtained gene chip data GSE13597 and GSE34573. GSE13597 is based on GPL570 platform (Affymetrix Human Genome U133 Plus 2.0 Array), and GSE34573 is based on GPL76 platform (Affymetrix Human Genome U133A Array). GSE13597 consisted of 25 NPC specimens and 3 normal specimens, while GSE34573 included 3 NPC specimens and 3 normal specimens.

The article "Identification of Key Genes in Nasopharyngeal Carcinoma Based on Bioinformatics Analysis" was retracted in 2023. Reasons: signs of a paper mill; compromised peer review; unreliable results or conclusions.

### 2.2. Identification of DEGs

Firstly, we used GEO2R tool to analyze microarray data GSE13597 and GSE34573 related to nasopharyngeal carcinoma. Volcano plot was generated using Bioconductor (https://bioconductor.org/biocLite.R). The “pheatmap” package in the R statistical software was used to draw heatmaps based on the top 10 regulated genes of GSE13597 and GSE34573.

### 2.3. GO and KEGG Analysis

GO and KEGG analyses were conducted via online tool DAVID (https://david.ncifcrf.gov/tools.jsp), and *P* value <0.05 was used as the critical value for screening significantly enriched genes. In this study, the main functions of DEGs were analyzed by “clusterprofiler” package in the R software.

### 2.4. Integration of PPI Network

To study molecular mechanism of nasopharyngeal carcinoma cell development and pathogenesis, we uploaded the DEGs of nasopharyngeal carcinoma to STRING (https://string-db.org/) software and applied Cytoscape software to draw PPI of DEGs.

## 3. Results

### 3.1. Identification of DEGs

GSE13597 and GSE34573 were analyzed online by GEO2R. 216 DEGs were obtained in GSE13597 between patient and control group (111 up-regulated DEGs and 105 down-regulated DEGs) (Figure 1(a)). 1101 DEGs were obtained in GSE34573 (470 up-regulated DEGs and 641 down-regulated DEGs) (Figure 1(b)). 63 common differential genes were screened named co-DEGs in the two datasets. We generated the heatmap of the top 10 NPC-related genes in the GSE13597 (Figure 2(a)) and GSE34573 (Figure 2(b)).

### 3.2. GO Annotation Analyses of DEGs

The DEGs of GSE13597 were associated with antimicrobial humoral response, defense response to bacterium, cell-matrix adhesion, tissue homeostasis, negative regulation of response to wounding, anatomical structure homeostasis, and humoral immune response. GO analysis revealed the DEGs of GSE34573 associated with cilium movement, microtubule-based movement, cilium organization, axoneme assembly, cilium assembly, microtubule bundle formation, and motile cilium assembly (Figure 3(b)). GO analysis of co-DEGs revealed the co-DEGs participated in leukocyte migration, positive regulation of kinase activity and MAPK cascade, cell chemotaxis, and myeloid leukocyte migration (Figure 3(c)).

The DEGs screened from GSE13597 relevant to NPC were related to chemokine signaling pathway, cell cycle, p53 signaling pathway, salivary secretion, complement and coagulation cascades, and IL-17 signaling pathway (Figure 4(a)). KEGG pathway analysis demonstrated that DEGs of GSE34573 were relevant to tyrosine metabolism, phenylalanine metabolism, histidine metabolism, glycerolipid metabolism, focal adhesion, and ECM-receptor interaction (Figure 4(b)). KEGG pathway analysis revealed that co-DEGs were relevant to IL-17 signaling pathway (Figure 4(c)).

The article "Identification of Key Genes in Nasopharyngeal Carcinoma Based on Bioinformatics Analysis" was retracted in 2023. Reasons: signs of a paper mill; compromised peer review; unreliable results or conclusions.

### 3.3. PPI Network and Hub Genes

We submitted 216 genes of GSE13597 and 299 genes of GSE34573 to STRING for PPI analysis, respectively, and identified seven hub genes, including FN1, MMP-10, MUC1, KIF23, CDK1, MUC5B, and MUC5AC (Figures 5(a)–5(i)).

## 4. Discussion

Despite the progress of radiotherapy technology, distant metastasis is still the main cause of treatment failure of NPC. Finding more effective treatment to reduce distant metastasis has attracted great attention. Therefore, understanding the etiology and mechanism of NPC progression is very important to improve survival and prevent NPC. In recent years, bioinformatics technology makes it easier for researchers to detect tumor gene changes on a large scale and has been widely used in the research field of major tumors.

We screened 216 and 1101 DEGs from GSE13597 and GSE34573 datasets, respectively. These DEGs were associated with chemokine-mediated signaling pathway, cell-matrix adhesion, tissue homeostasis, defense response to bacterium, humoral immune response, cilium movement, cilium organization, cilium assembly, and epithelial cilium movement. In addition, DEGs were relevant to p53 signaling pathway, salivary secretion, complement and coagulation cascades, and IL-17 signaling pathway. The functional defects of cell cycle and cell proliferation regulators participated in the development and progression of tumor cell. Based on PPI network, seven hub genes that can deeply understand the pathogenesis of NPC at the molecular level are obtained, including FN1, MMP-10, MUC1, KIF23, CDK1, MUC5B, and MUC5AC. Xi et al. selected four genes including CRIP1, KITLG, MARK1, and PGAP1 as candidate genes affecting nasopharyngeal carcinoma-based gene expression profile analysis [4].

Fibronectin-1 (FN1) is a member of the FN family, which was confirmed to be associated with EMT, which could enhance cancer cell invasion and metastasis [5, 6]. FN1 was up-regulated in many human tumors such as breast cancer and colorectal cancer and was involved in tumor regulation [7, 9]. FN1 was higher expressed in papillary thyroid cancer tissues, and knockout of FN1 suppressed the proliferation and adhesion of papillary thyroid cancer cell [10]. Degradation of extracellular matrix components mediated via matrix metalloproteinases (MMPs) is a necessary step for the invasion and metastasis of cancer cells. MMP-10 is an important member of MMPs. MMP-10 was anomalously expressed in numerous tumors, such as gastric cancer [11], esophageal cancer [12], and head and neck cancer [13]. MMP-10 is a protease closely related to tumor invasion and metastasis, whose main function is to degrade extracellular matrix. MMP-10 can destroy the physical barrier around tumor cells and reduce the adhesion between tumor cells, so as to make tumor cells grow around. MMP-10 can also promote the formation of tumor blood vessels through the reconstruction of basement membrane, so as to promote the proliferation and metastasis of malignant tumor cells. Therefore, MMP-10 is a promoter of tumor invasion and metastasis.

The article "Identification of Key Genes in Nasopharyngeal Carcinoma Based on Bioinformatics Analysis" was retracted in 2023. Reasons: signs of a paper mill; compromised peer review; unreliable results or conclusions.

MUC1 is a high molecular weight mucin rich in serine, threonine, and proline enzymes. MUC1 is anomalously expressed in numerous cancers. The coding production of MUC1 gene was a tumor marker for the diagnosis of thyroid cancer [14, 15]. MUC1 expression is reported to be an important molecular marker of cervical squamous cell carcinoma [16]. Numerous studies confirmed that MUC1 can enhance the proliferation and metastasis of different tumor cells [17–19]. The cytoplasmic end of MUC1 can be used as a scaffold to activate multiple signal pathways through the activation of specific kinases, including PI3K, Akt, and MAPK [20–22]. These signal pathways can enhance cell differentiation and proliferation and regulate the expression of adhesion molecules. As a member of the KIF family, KIF23 plays the role of a molecular motor. It is an ortho-end-directed motor enzyme that moves antiparallel microtubules in vitro and plays an important role in the bundling and transport of microtubules at specific locations and times in different types of cells. KIF23 is a key regulator of cytokinesis and may become a therapeutic target for many diseases in the future. KIF23 is highly expressed in a variety of malignant tumors, promotes cell proliferation, and is related to poor survival and poor clinicopathological features [23].

Hoshi et al. interfered with the expression of MUC5AC by small RNA technology and found that MUC5AC knockout in vivo inhibited the proliferation and migration of pancreatic cancer [24]. Inaguma et al. found that overexpression of MUC5AC interferes with the membrane localization of E-calcium protein, thereby reducing the adhesion of E-dependent calcium protein cells and promoting the invasion and migration of pancreatic cancer cells [25]. Hoshi et al. found that the expression of MUC5AC was higher in pancreatic cancer cells and MUC5AC inhibited IL-6 expression and TRAIL signaling pathway to inhibit the migration of neutrophils [24].

CDKs belong to serine/threonine kinases, which play a role in all stages of the cell cycle and promote the orderly proliferation of cells [26]. Abnormal regulation of cell cycle is one of the important reasons for tumor cell proliferation. As an important factor in cell cycle regulation, cyclin dependent kinases (CDKs) are highly expressed in many tumors, resulting in abnormal cell cycle. Based on the bioinformatics study, Dong et al. found that some genes including CDK1 were relevant to the prognosis of pancreatic cancer [27]. Piao et al. found that CDK1 was overexpressed in pancreatic cancer and the expression of CDK1 was relevant to histological grade, tumor size, and survival time of pancreatic cancer patients [28].

The article "Identification of Key Genes in Nasopharyngeal Carcinoma Based on Bioinformatics Analysis" was retracted in 2023. Reasons: signs of a paper mill; compromised peer review; unreliable results or conclusions.

In conclusion, seven hub genes, including FN1, MMP-10, MUC1, KIF23, CDK1, MUC5B, and MUC5AC, might be therapeutic potential biomarkers of NPC.

## Figures and Tables

**Figure 1:** Volcano plots of DEGs in GSE13597 (a) and GSE34573 (b).

**Figure 2:** The heatmap plots of the top 10 genes. (a) GSE13597. (b) GSE34573.

**Figure 3:** Gene ontology (GO) analyses of DEGs. (a) GO analysis of DEGs of GSE13597. (b) GO analysis of DEGs of GSE34573. (c) GO analysis of co-DEGs of GSE13597 and GSE34573. KEGG pathway enrichment analyses of DEGs.

**Figure 4:** KEGG analyses of DEGs. (a) GSE13597. (b) GSE34573. (c) Co-DEGs of GSE13597 and GSE34573.

**Figure 5:** PPI networks based on the screened DEGs. (a–c) GSE13597. (d–f) GSE34573. (g–i) co-DEGs of GSE13597 and GSE34573.

## Data Availability

Data used to support the findings of this study are available on reasonable request from the corresponding author.
